# Restaurant Interior Design under Digital Image Processing Based on Visual Sensing Technology

**DOI:** 10.1155/2022/3302700

**Published:** 2022-06-08

**Authors:** Yan Wan, Can Cui, Guanqiang Wang

**Affiliations:** Faculty of Humanities and Arts, Macau University of Science and Technology, Avenida Wai Long, Taipa 999078, Macau, China

## Abstract

With the development of the social economy, people are paying more and more attention to decorative effects and the comfort and individual characteristics of decoration. To meet the increasingly high requirements of customers, many restaurants have begun to focus on the personalization of the dining environment, which is comfortable to build and focuses on the spiritual satisfaction and experience of customers during the dining process. In this study, a comprehensive analysis of digital image processing technology is performed to implement an automatic illumination system with improved performance for the restaurant interior design and embed the restaurant interior design with intelligence. The convolutional neural network (CNN) is employed in the automatic illumination system to develop the human body recognition model. After a test of its recognition accuracy, the parameters of CNN are optimized, and high recognition accuracy of 0.97 is achieved. Compared with other models, the process of training the designed model implemented in this study can finish in 40 minutes, and the performance has been well optimized. Moreover, the processing function of the model is also able to resist the interference of other external objects. The excellent automatic illuminating system can greatly improve the atmosphere as well as the service level of the restaurant at night, which can promote the modernization of the restaurant and give certain reference significance to the reform and advancement of the decoration industry.

## 1. Introduction

With the advancement of social science, technology, and economy, modern customers place a high value on the entire level of restaurant facilities when selecting a restaurant. The night is the main working time of the catering service industry, and the illuminating system has a great impact on the service and convenience for both customers and the staff of the restaurants [1]. From the perspective of the decoration design, the design of the illuminating system needs to be fully considered by the managers of restaurants. However, the traditional illuminating system is disturbed by the external environment. In the past, the illuminating cannot be controlled accurately due to the diversity of human factors, such as staff forgetting to turn off the light and other forms of waste on the electricity power. Visual sensing is used in a variety of disciplines to generate ideas for restaurant interior design lighting. As a result, the emphasis is on improving the system's digital image processing capability and optimizing the illuminating system [2].

At present, illuminating control technology is generally divided into remote control, automatic physical sensor control, and machine vision control embedded with artificial intelligence (AI) [3]. Previously, physical sensors were used for illuminating control, which liberated people's hands. However, in this process, under the control of physical sensors, the final decision of the illuminating system will sometimes be against people's original intention [4]. For example, the monitoring index without an infrared sensor is to detect the movement of objects, but the environment is complex, and these simple inferences are not particularly accurate. Inspired by computer technologies and the improvement of deep learning (DL) theory, scholars found that machine vision technology (VT) has a good improvement in data and image recognition and is the most potential control technology in the future. Generally, machine VT is superior to manual operation in many aspects. The most widely used technical scheme is recognition based on machine learning techniques such as DL [5]. Compared with manual modeling, the model can automatically fit the characteristics of the recognition area [6]. In the manual modeling recognition scheme, the recognition scheme will be disturbed by many aspects such as target size. For example, if the size of the recognized object is too large, the model will be confused with the target object, and the recognition accuracy will be seriously disturbed.

Wan [7] created the influence model of user consumption behavior and selected statistical indicators to finish the research process based on evaluating user consumption behavior patterns and defining factors affecting consumer behavior. The simulation experiment demonstrated that the method's study results can be used to improve restaurant operations and have practical relevance. Literature [8] mentioned the approach of consumer behavior influence analysis utilizing LMDI theory, which entails evaluating a significant amount of data and then studying the influence of connected aspects by extracting the data's core laws and features. When this influence analysis method is applied to the subject of restaurant interior design as a research object, it not only has requirements for the comprehensiveness and objectivity of data processing and the method of data inclusion laws processing, but also has more stringent criteria for data sources, resulting in more limitations and poor results. The analysis approach described in [9] is too subjective in terms of selecting impact analysis-related indicators and selecting analysis components to reach the desired outcomes. Bo and Haung [10] investigated the fundamental theory of image style transfer using image style transfer technology, Gram matrix, and Poisson image editing technology, as well as image segmentation, content loss, enhanced style loss, and Poisson image editing constrained picture spatial gradient. Chen and Mang [11] created an interactive device that may be used to divert customers' attention while they wait and allow them to enjoy the excitement of using it, thereby assisting restaurant owners in promoting their garden restaurants and local postcards. To propose the design idea of the interactive gadget, a literature review on human-computer interaction, wearable devices, and generative art was conducted. Furthermore, prototypes, a user manual, and user suggestions were created, and the prototype's effectiveness was evaluated. Warakul and Vorapat [12] investigated the relationship between emotional responses to interior color and restaurant decisions. A total of 496 research participants evaluated eleven computer-generated restaurant settings with varying interior colors. Each participant was asked to rate his or her emotional responses on the PAD emotion scale's nine adjective pairs, as well as their decision to enter the study. The chance of attending the restaurant was calculated using logistic regression models. The pleasure was discovered to be the most accurate predictor of behavioral responses.

To implement a better performing illuminating control system for restaurant interior design using visual sensing technology, a detailed analysis of the principle of digital image processing technology is performed, and then a design with the human body recognition model is proposed using CNN, which gives an order to the illuminating system to control the switch of the lights. After a test of its recognition accuracy, the parameters of CNN are optimized, and high recognition accuracy of 0.97 is achieved. It is found that the human body recognition model designed here has been improved, and the processing results of digital images have been optimized. Using this human recognition model, the service level of the restaurant at night can be largely improved, which is of great significance to the development of the modern design concept of the restaurant.

The rest of the manuscript is organized into 3 sections. In Section 2, a detailed description of the proposed method is presented and artificial neural network and convolution neural network are illustrated.  Section 3 illustrates the results obtained with the proposed model, and Section 4 concludes the manuscript.

## 2. Materials and Methods

### 2.1. Storage Mode of Digital Image

Generally, the optical image must be transformed to a digital image before the image captured by the camera in electronic equipment may be saved effectively. The processing of images is based on the storage of collected images. Normally, bitmap storage discretizes the image into many pixels, and the color data are separated by channels. The image will be retained in the disk in the state of the matrix [13]. The number of rows and columns of the matrix represents the pixel length and width of the retained image, and the corresponding coordinate data represents the pixel value of the image. Different pictures may have differences in their quality. Therefore, there are differences in the values of pixels, most of which are 8-bit, 16-bit, and 24-bit color resolutions. In a practical scenario, people prefer to choose 8-bit color resolution, which can discretize the color into a number among [0, 25]. Generally, pixel images can be divided into two types based on the number of channels, one is a single channel gray image, which generally contains black-and-white photos, and the other is a multichannel color image [14]. As for the storage mode of a single channel gray image, the row and column coordinates of the image matrix will correspond to the corresponding pixel values, and the pixel values represent the depth of the image itself. For example, when the color resolution is 8 bits, the color discrete interval is a constant among [0, 25]; the smaller the color dispersion, the more obvious the black degree of the image itself, and the larger the color dispersion, the whiter the image itself. If the value is in the middle, it represents the gray value that gradually changes according to the numerical ratio. In a multichannel color image, if the image color resolution is 8 bits, there are three channels, and the coordinate values of each row and column of the image matrix are corresponding, and the three-pixel values, in turn, correspond to the gray values of red, green, and blue. For example, in a channel, 0 represents that there is no blue, and the corresponding 255 means the picture is the bluest, and it is the same for other channels. Therefore, the overall color of the image is the effect of the combination of the gray values of the three channels [15].

In the image process, Fourier transform is used to transfer the signal from the time domain to the frequency domain and process the signal in the frequency domain, to analyze the composition of signal frequency more accurately, and to lay the foundation for filtering operation. In the section of image processing, after the Fourier transform of an image, the image is transferred from the spatial domain to the frequency domain. Therefore, the Fourier operation is performed on the image. It is roughly the basis of image feature extraction and the basic and necessary conditions of image edge detection and filtering noise reduction. If the pixel size of an image is specified as *M∗N*, (1) can be obtained as a two-dimensional Fourier transform:

(1) $$\begin{array}{c} F\left(\mu ,\theta \right)=\sum_{x=0}^{M-1}\sum_{y=1}^{N-1}f\left(x,y\right)e^{-i2\pi \left(\mu x/M+\theta y/N\right)}, \end{array}$$

where *f*(*x*, *y*) represents the row and column pixels in the spatial domain and *F*(*μ*, *θ*) denotes the value of the frequency domain obtained after Fourier processing, which is expressed in the form of a complex number. Conversion helps to obtain all the information of the image included in the frequency spectrum. However, only the amplitude spectrum is used in frequency analysis [16]. Parameters *R* and *I* are used to express the real and imaginary parts of the image and that need to be supplemented in the *F*(*μ*, *θ*). Equation (2) demonstrates the amplitude spectrum of the image.

(2) $$\begin{array}{c} \left|F\left(\mu ,\theta \right)\right|=\sqrt{R{\left(\mu ,\theta \right)}^{2}+I{\left(\mu ,\theta \right)}^{2}}. \end{array}$$

After the amplitude spectrum is obtained, the frequency of the image can be displayed on the complex coordinates. In the field of a digital image, the spatial frequency represents the frequency of periodic change of image gray within the correlation distance, which reflects whether the change of pixel value is obvious, that is, the gradient of the pixel value in the plane space. When analyzing the amplitude spectrum, if there are more high frequencies, it indicates that the overall fineness of the image is positively correlated with the interference component. On the contrary, if there are many low-frequency components, the smoothness of the image is negatively correlated with the interference component.

### 2.2. Equalization of the Histogram of Image and Processing of Image Pyramid

In the process of image acquisition, shooting is a crucial element of the picture acquisition process and is frequently disrupted by unsteady illumination and aberrant sensors, resulting in varying image capture times and changes in image brightness and color balance. As a result of the ongoing research into graphics processing, scholars have discovered a histogram equalization approach that reduces the impact of external light on the image [17]. Furthermore, it can also repair underexposed and overexposed images. Histogram equalization can also be called histogram flattening. If the brightness range of the initial image is very small and the contrast is not very good, histogram equalization can play a role in visual enhancement. This method is suitable for images with locally high or low brightness, which is of relatively good effect [18].

In the process of image processing, the image size is often adjusted and changed. In the specific operation, the original size of the image will be enlarged or reduced. In essence, the image is sampled up or down. Hence, the image pyramid is a sampling method. It is called an image pyramid, because at the beginning when an image is sampled up or down, it forms a set of atlases. In these atlases, it covers images under various scales. The bottom of the pyramid is the largest scale and the smallest scale at the top. Through the aforementioned steps, a pyramid-like structure is constructed. Not only can the size of the images be adjusted, but also the image features may be retrieved when the images are sampled up or down, to obtain the features in various “depth of field” states [16]. It is like the visual effect of people observing the size of the object.  Figure 1 demonstrates the structure of the “image pyramid.”

Generally, two common methods are used to build image pyramids: one is the Gaussian pyramid, and the other is Plath pyramid [19]. The former is generally used in the downsampling of the image to reduce the size of the image, while the latter is generally used when the image size changes, to repair the original image as much as possible. Gaussian pyramid is used to perform Gaussian blur processing on the image and then downsampling. Because the direction of Gaussian convolution kernels is the same, there is generally no other noise with Gaussian blur, so it is widely used. There are generally two important steps in the construction of the Gaussian pyramid. First, Gaussian blur processing must be carried out on the image; that is, the Gaussian convolution kernel and the initial image function convolution processing need to be used to obtain the blurred image. Then, in the downsampling operation of the blurred image, generally, the odd and even rows of image pixels can be deleted. After these two steps, the first layer of the Gaussian pyramid appears. The specific number of layers can be changed according to the actual situation, and there is no fixed level. When the Laplacian pyramid samples the image upward [20], it needs to be used in combination with the Gaussian pyramid, and the first related sampling process also needs two steps. Primarily, the number of image pixels should be in the row and column, which is expanded twice in the direction, which is generally realized by adding pixel values on the odd and even rows. Afterward, the expanded image needs to be processed by Gaussian blur, and the pixel value added to the row should be given a new value. Generally, the image sampled upward will be unclear. The reason for this is that after sampling, some information in the image is lost, and the Laplace pyramid can record the lost information so that the lost information of the image can be better recorded. Equation (3) illustrates the construction of layer I of the Laplace pyramid.

(3) $$\begin{array}{c} L_{i}=G_{i}-UP\left(G_{i+1}\right)⊗\varsigma_{5\times 5}, \end{array}$$

where *G*_*i*_ represents the image of layer *i* of the Gaussian pyramid, *UP*(*G*_*i*+*l*_) means the sampling of the image of *i* + 1*th* layer of the Gaussian pyramid, and *ς*_5×5_ refers to the 5 × 5 Gaussian convolution kernel. Therefore, the Laplacian pyramid essentially retains the data residuals between different layers of the Gaussian pyramid.

### 2.3. Application of Neural Network in Image Processing

The neural network model is frequently used in the field of AI, which contributes a reliable theoretical basis to DL. It is inspired by the model of human brain neurons receiving, summarizing, and outputting information [21]. To more clearly understand the relatively complete DL neural network model, it is necessary to understand the core content of its basic artificial neural network, mainly from several aspects as shown in Figure 2.

The following is a systematic description of the neuron structure, neural network topology, and neural network selection weights to learn algorithms.

#### 2.3.1. Neuron Structure

The components of biological neurons mainly include several parts as shown in Figure 3.

Among the relevant elements mentioned in Figure 3, dendrites can be regarded as the input of neurons, which are used to access the charge signals transmitted by other cells. Axons can be regarded as the output of neurons, which transmit the charge signals to relevant cells, and synapses are used as the input and output ports, which generally play the function of connecting neurons so that neurons can contact multiple neurons. There is membrane potential in the cell body. The charge signal from the outside alters the membrane potential and causes it to rise continuously. When the membrane potential rises to exceed the relevant threshold, the neuron will activate, generate a pulse, and transmit it to the next neuron [22]. The conversion between input and output of neural network system is generally expressed in graphics, and a single neuron can be represented by a single neuron model structure as shown in Figure 4.

In the single neuron model structure, the neuron input vector is expressed in matrix form, and the weight matrix is expressed as follows:

(4) $$\begin{array}{c} Y={\left[y_{1}y_{\ldots }y_{r}\right]}^{T},\\ W={\left[w_{1}w_{\ldots }w_{r}\right]}^{T}. \end{array}$$

*Y* represents the axon information of relevant neurons, *W* denotes the relevant information transmission efficiency of synapses, and the corresponding relationship between the output *Z* of one neuron and the input P of the other can be expressed as

(5) $$\begin{array}{c} Z=f\left(\sum_{j=1}^{r}w_{j}y_{j}+c\right)=f\left(W\times Y+c\right). \end{array}$$

The parameter *c* in (5) stands for the threshold or deviation, and *f* points to the relevant activation function.

#### 2.3.2. Neural Network Topology

Generally known topologies of the neural network include single-layer feedforward networks, multilayer feedforward networks, feedback networks, stochastic neural networks, and competitive neural networks [23].

#### 2.3.3. Neural Networks Weights and Learning Algorithms

Learning in neural networks is generally called training. Through the influence of the relevant conditions of neural networks, the relevant connection weights are adjusted for neural networks, so that neural networks can respond to the external environment in different ways. Different neural networks have relevant activation functions and specific roots which are adjusted according to the specific situation, which is generally recorded as *y*=*f*(*x*); the training process is to use the given data *x* and *y* to fit the activation function *F*. The training of neural networks can be divided into two types: one is tutor learning and the other is nontutor learning. There is expected output in tutor learning. After adjusting the weight, the predicted relevant output can be close to the expected output to the greatest extent while there is no tutor. The learning gives the measurement scale representing the quality of the method, and the parameters are processed according to this scale.

### 2.4. Design of CNN

With the continuous improvement of social science and technology levels, restaurant consumption is gradually a kind of unavoidable consumption for the majority of consumers. People's expectations for restaurant decoration have gradually increased as the service style, features, quality, and other aspects of the social catering business have improved. Good decoration and decoration in line with people's expectations can attract consumers to consume. There are many theoretical models in deep learning. Usually, the CNN is selected as the model for recognition to integrate the intelligent concept into the interior decoration of the restaurant, when the illuminating system restaurant interior design is being implemented [24]. Next, the visual sensing of illuminating is constructed based on CNN. The layers of the CNN model include the output layer, convolution layer, pooling layer, and full connection layer.  Figure 5 displays the structure of a common CNN.

In CNN, the convolution layer generally uses the convolution kernel and the input image for convolution operation.  Figure 6 demonstrates the structure of the convolution kernel.

If the image is treated as a complete individual for feature extraction and fitting during image processing during convolution, it is usually because the target in the image is too small and there is too much background and other interference, preventing the training data from fitting due to background differences. The convolution layer uses the provided size. The image features can be obtained from local to global when the convolution kernel is used for convolution, avoiding the disadvantage of a significant amount of computation when obtaining the features from the entire image. The resulting features will become increasingly abstract as the number of layers is increased [25].

After convolution, the pooling layer is generally used which uses the output of the convolution layer as input. The main difference between the pooling layer and the convolution layer is the number of domain operators used by the pooling layer and convolution layer. Specifically, the purpose of the convolution layer is to obtain the local feature data of the image, and the purpose of the pooling layer is to sample the image, reduce the size of the image, and reduce the amount of information to be processed by the next layer. Additionally, it can make the volume of the next layer. The integrable layer can obtain the image feature data from the whole so that the CNN has the feature extraction logic from local to the whole.

### 2.5. Implementation of CNN

When building a new CNN model, a lot of training datasets and related interference datasets for model training are usually required. In the study, CNN is employed to design a relatively excellent illuminating system in the restaurant, so there is a need to identify the human body in the environment. Therefore, the training datasets and interference datasets are based on image data. In the process of CNN model training, if too much data is loaded at one time, it will occupy more memory and make the training process very lasting. If the intermediate program is abnormal, all previous efforts will be wasted. To reduce the training cost, while training CNN, it is necessary to be between the amount of data and the number of training time to find a balance point, to reduce the amount of image data in a certain time and increase the number of programs training [26]. In the present study, the size of the image is defined as 224*∗*224 pixels, and the CNN model is designed using this format. When there are more than two layers of CNN, the continuous curve can be fitted in two-dimensional space, and it should cooperate with relevant nonlinear activation functions because the high-dimensional space fitting problem will be designed in the process of image classification and recognition. In the proposed CNN model, the lowest three-layer CNN model is used to construct the human body recognition model. When the convolution kernel size is 1*∗*1, it is difficult for the convolution kernel to capture the image features. Therefore, the size of the convolution kernel employed is 3*∗*3. When the connection layer is established, all the matrix characteristic data are converted into a one-dimensional row vector. After 1D vector operation, the amount of data in the one-dimensional row vector is reduced to 1024, and then the ReLU.

The activation function is used for nonlinear operation. The relevant row vectors are obtained after performing a vector operation on all of the feature data. The row vectors are utilized to express the quantitative relationship of the corresponding categorization throughout the training. The CNN model is depicted in Figure 7.

### 2.6. Case Analysis

The training image data for the model developed in this study is derived from actual life, including image data of human activities and trivial life. The training set consists of 1200 human images, whereas the interference dataset consists of 1000 human activity images. To better evaluate the accuracy of the CNN model, additional 400 processed human activities and other images are used in the evaluation of the model. The camera utilized in this experiment is a Raspberry Pi device. The selected camera has 5 million pixels and can record images with a resolution of 2592*∗*1944.  Figure 8 presents the camera.

After the model training is completed, the recognition accuracy of the model is tested, and the performance is compared with the famous “Cats VS Dogs” model.

## 3. Results

### 3.1. Human Body Recognition Model Recognition Accuracy Test

CNN has become the go-to model for any image-related issue. It outperforms the competitors in terms of accuracy. It is also used in recommender systems, natural language processing, and other areas. The fundamental advantage of CNN over its predecessors is that it discovers important features without the need for human intervention. In addition, CNN is computationally efficient. It performs parameter sharing and uses special convolution and pooling algorithms. CNN models can now run on any device, making them globally appealing.  Figure 9 manifests the CNN accuracy for the human recognition model in a restaurant using the additional 400 test images after training.

When the CNN model is trained for 500s, the model recognition accuracy can reach a maximum of 0.978, according to the accuracy test of the constructed human body recognition model. The model recognition accuracy can reach 0.973 when the training reaches the 2000s. This indicates that the model's maximum stable recognition accuracy is 0.973. The high performance of CNN is due to its strength for implicit feature extraction. The spatial features are extracted from image input when CNN is used. When thousands of features need to be extracted, CNN is suitable. CNN collects these features on its own rather than having to measure each one individually.

### 3.2. Comprehensive Performance Test of Human Recognition Model

The model effect of “Cats VS Dogs” trained on 25000 pictures is compared with the proposed human recognition model trained on 2200 pictures. The comparative results are shown in Figure 10.

After comparing with the Cats VS Dogs model, it is found that the proposed restaurant model has achieved 97% recognition accuracy in only 40 minutes, indicating that after the optimization of the designed human body recognition model, the cost of the final visual sensing system has been controlled and can meet the practical need of the illumination system of the restaurant. The application of the model in the decoration of the restaurant can well improve the overall environmental conditions of the restaurant.

## 4. Conclusion

With the development of economic level, when people choose restaurants, they often have high requirements for the overall facility level of restaurants. The night is the key working time of the catering service industry, and the illuminating system has a great impact on it. The illumination system has a significant impact on the restaurant service's critical working hours, which is at night. The design of the illumination system must be completely considered in the decorative design. To integrate the intelligence concept into the illuminating system of restaurant interior design, the human body recognition model in the illuminating system is constructed based on the CNN. By optimizing the parameters of the CNN, the recognition efficiency and accuracy of the human body recognition model based on the CNN are effectively strengthened. The accuracy of the model has been improved significantly, which strengthens the processing ability of digital images and can resist the interference of other external objects. In comparison to previous models, the training process for the proposed model used in this study may be completed in 40 minutes, and the performance has been well optimized. The proposed illumination system can substantially improve the restaurant's atmosphere as well as service level at night, promoting restaurant modernization.

## Figures and Tables

**Figure 1:** Structure of image pyramid.

**Figure 2:** The core content of artificial neural network.

**Figure 3:** Composition of biological neurons.

**Figure 4:** Single neuron model structure.

**Figure 5:** CNN structure.

**Figure 6:** Structure of convolution kernel.

**Figure 7:** Structure of CNN model.

**Figure 8:** Raspberry Pi.

**Figure 9:** Accuracy test of the human body recognition model.

**Figure 10:** Performance comparison of different models: (a) Cats VS Dogs and (b) human body recognition model.

## Data Availability

The data used to support the findings of this study are available from the corresponding author upon request.
